# Impact of *Status quo* and Resistance to Innovation on the Failure of Detection and Prevention Strategies of Drugs Control Committee in Malaysia

**DOI:** 10.3389/fpsyg.2022.922785

**Published:** 2022-06-21

**Authors:** Zhen Zeng

**Affiliations:** Guangxi Police College, Nanning, China

**Keywords:** *status quo*, resistance to the innovative nature, drug control committee, failure of detection and prevention strategies, poor team performance

## Abstract

The detection and prevention strategies for drug control have gained significant attention from the drug control committees globally and need the researchers’ attention to improve these strategies worldwide. Hence, this research investigates the impact of the *status quo* (SQ) and resistance to the innovative nature of the drug control committee on the failure of detection and prevention strategies (FDPS) in Malaysia. This article also analyzes the mediating role of poor team performance (PTP) among the SQ and resistance to the innovative nature of the drug control committee and the FDPS in Malaysia. This study has employed the primary data collection ways such as questionnaires to gather the data from selected respondents. The researchers also applied the SPSS-AMOS to check the association among variables and testing of hypotheses. The results revealed that the SQ and resistance to the innovative nature of the drug control committee have a positive association with the FDPS in Malaysia. The findings have also exposed that PTP significantly mediates between the SQ and resistance to the innovative nature of the drug control committee and the FDPS in Malaysia. This study guides the policymakers that they should develop the policies that eliminate the SQ nature and motivate the committee to adopt innovations that enhance the team performance and success of detection and prevention strategies in Malaysia.

## Introduction

Malaysia, a developing country in Southeast Asia, has a national pharmacovigilance center, the “National Adverse Drug Reaction Monitoring Centre,” which serves the whole country. Certain big hospitals and pharmaceutical firms use adverse drug reaction (ADR) monitoring systems, but the national center consolidates all of their findings. Doctors, pharmacists, and dentists often complete reports voluntarily. However, marketing authorization holders are required to submit reports. These individuals watch human-use pharmaceuticals, vaccines, and biological and herbal therapies. The National Drug Reaction (ADR) Center employs monthly updated prepaid postage report forms or report cards. An advisory group at the national center evaluates the casualties documented in the ADRs. The Drug Control Authority (DCA) created the Malaysian Adverse Drug Reaction Advisory Committee (MADRAC) to assess the safety profiles of medications authorized for use in Malaysia. The DCA receives drug safety information from MADRAC both locally and abroad (Mardian et al., 2021).

In 1990, the National Drug Safety Monitoring Centre, which serves as MADRAC’s secretariat, was recognized as the World Health Organization’s (WHO) Safety Monitoring Program’s 30th member. All ADR reports collected and vetted by MADRAC are sent to the Uppsala Monitoring Centre in Sweden for inclusion in the WHO database. MADRAC also encourages ADR reporting in Malaysia and provides information and advice to the DCA so that regulatory action may be taken in response to ADRs received locally and globally. It also participates in the WHO ADR monitoring program and offers ADR information to doctors, pharmacists, and other healthcare providers. Malaysia’s present medication safety system has limitations (Rodzlan Hasani et al., 2019), namely, (1) in terms of pharmaceutical vigilance, there is a lack of understanding concerning medication safety among healthcare workers, (2) there is a lack of understanding regarding the presence, function, and purpose of national ADR reporting (Shafie et al., 2019), (3) due to the lack of a national computerized database on the prescription administered, signal production is difficult, (4) inability to engage pharmaceutical companies with drug safety issues, (5) there is a lack of knowledge on genetic effects, social behaviors, pharmacological interactions, and contraindications linked with medicines, (6) only a few reports on traditional and herbal medications, which are commonly utilized, are present, (7) underreporting is a key flaw in all spontaneous reporting systems, (8) nursing personnel and customers were not involved in the ADR monitoring program, (9) the role of nongovernmental organizations (NGOs) in drug safety problems is limited, (10) the function of the media in public drug safety education is limited, (11) healthcare practitioners’ selective reporting (reporting bias), and (12) inadequate at spotting delayed ADRs. These limitations play a vital role in the success or failure of the policies related to the prevention and control of drugs in Malaysia. This is why this study aimed to investigate the reason for the failure of prevention and control of drug-related strategies in Malaysia. The value of Pharma products exported from Malaysia (million US$) is given in Figure 1.

**FIGURE 1:** The value of Pharma products exported from Malaysia.

The detection and prevention strategies for drug control have gained significant attention due to the high rate of drugs addiction around the globe and need the researchers’ attention to improve these strategies worldwide. In addition, the drug addiction situation has also gained an increasing trend with time in Malaysia, and this situation also motivates the researcher to examine the drug control committee strategies to control this situation in the country. Moreover, significant regulations are needed for the control of drug addiction in the country, and for the regulators’ guidance, there is a need to examine drug control committee strategies to help the regulators in developing regulations. All of these situations motivate the researchers to look into this area and investigate the impact of the *status quo* (SQ) and resistance to the innovative nature of the drug control committee on the failure of detection and prevention strategies (FDPS) and also analyze the mediating role of poor team performance (PTP) among the SQ and resistance to the innovative nature of the drug control committee and the FDPS in Malaysia. The significance of the study is (1) it will highlight the importance of drug prevention strategies in Malaysia, (2) it will help pharmaceutical industry-related professionals revamp their policies to support and composition of better policies and strategies for drugs in Malaysia, and (3) it will help the researchers to identify and explore the more horizon of drug prevention and control strategies in Malaysia.

The study structure is divided into five phases. The first phase presents the introduction. In the second phase of the study, the pieces of evidence regarding SQ nature, resistance to innovative nature (RTIN), PTP, and FDPS are discussed in the light of past literature. The third phase of the study shines the spotlight on the methodology employed for collecting data regarding SQ nature, RTIN, PTP, and FDPS, and its validity is analyzed. In the fourth phase, the study results are compared with the pieces of evidence reviewed from the literature. In the last phase, the study implications and the conclusion and future recommendations are presented, concluding this article.

## Literature Review

This section of this article shows the literature related to the past studies about the understudy variables such as SQ, resistance to the innovative nature, FDPS, and PTP and subsections.

### *Status quo* and Failure of Detection and Prevention Strategies

From the past few years, the strategies or growth when restrains to move further and remains constant brings the eminence of SQ nature. The SQ is the current nature of affairs and observation of social, political, religious, or military issues. We live in a world where modern states are the SQ and remain on their rules and policies, such as Malaysia. Taylor and Cheng (2022) analyzed the matter of SQ that clearly influences the failure of prevention and detection strategies. Many people always want to maintain the SQ nature to maintain effective detection and prevention strategies. The SQ nature is a good thing for certain impacts on the FDPS. Turner and Nymalm (2019) enumerated the progress and morality of the SQ that builds a narrative over the strategies to be formed for the prevention of illegalities. According to sociological beliefs, the SQ nature assigns to the ongoing case of social system and beliefs in Malaysia. With the view of political argument, it measures how circumstances are contradictory with a desirable adjustment toward strategies. The countries, such as Malaysia, are currently demanding to control the SQ nature with respect to their nuclear arsenals. Liu (2021) examined the revisionism and SQ approaches over the projects established to control and prevent the drugs. Although improvements or changes can always be made and cannot be restrained at some stages, the SQ nature should be tested due to discrimination and causing impacts on the FDPS. Vinaik et al. (2019) explored the prevention and management of drugs that are usually SQ in nature. The SQ nature can be challenging to some countries, such as Malaysia, as it means running in contrast to the way conditions are presently being completed. The nature of the SQ is highly influential toward the failure of strategies that are being built by some developing as well as developed countries. Duke et al. (2020) assessed the criminal justice system that is responsible for the prevention and detection of drugs. In Malaysia, the policies and strategies are built in accordance with the threats to its economic and administrative forums. Therefore, the efficacious nature of the SQ not only prevents the threats but also helps the government to proceed toward the establishment of detection and prevention strategies.

**H1:** SQ nature significantly impacts the FDPS.

### Resistance to Innovation and Failure of Detection and Prevention Strategies

Resistance to change is the act of conflicting and excruciating adjustment and conversion of effective strategies for the world (Chien et al., 2021a). This resistance can manifest itself in one employee or in the workplace as a whole. Resistance to innovation is the unwillingness to adapt to a modified state of affairs, especially in Malaysia. Stryja and Satzger (2019) assessed the resistance toward innovation that is considered the main barrier to the development of detection and prevention strategies in controlling drugs. The resistance to innovation is an element that arises after the huge prevalence of criticism among people who are negative toward the detection and prevention of threats. Not only has this but the communities that are major barriers toward the innovation endorsed their sarcastic remarks on the strategies beneficial for the growth of a country. van der Merwe et al. (2020) explored the dynamics of resistance in innovation systems that are important functions in preventing the elements of controlling drugs. In Malaysia, many commitments are failed with the neighboring countries just due to the failed comments of people who are working against the policies of rising Malaysia. Ranci and Arlotti (2019) narrated the change and the resistance to it that is the main problem for the policy implementation for the controls of drugs. The continuous resistance toward innovation leads people toward the endless comments that are usually highlighted in the international forums. This damages the status of countries that are striving for better economic and innovative changes to lead their sectors better in a competitive world. Arena Ventura et al. (2019) discussed the prevention of drugs from the perspectives of users and families due to high consumption in the world. Managing the resistance to change is challenging for Malaysia and could result in the failure of implementing detection and prevention strategies. It is mindful that all the communities aren’t the reason behind any kind of resistance. Hence, the involvement of all communities in resistance toward the innovation can cause serious threats when governments continuously introduce change to your system. Rich (2020) enumerated the understanding and perspectives of drugs and their prevention according to the resistance to innovation. Systems and departments are constantly evolving, which means change is inevitable. However, introducing changes without consulting the people they affect, describing the need for change, and giving support through the process will alienate workers and drag down morale. When a change is introduced in an environment, with a lot of discussions and employee involvement, resistance to change is minimized.

**H2:** RTIN significantly impacts the FDPS.

### Mediating Impact of Poor Team Performance

The SQ is a passionate bias and a desire for the existing state of trading as well as establishing standards for detection and prevention strategies for drug controls. The existing SQ nature is seized as an allusion point, and any change from the control of drugs is anticipated as a loss without consulting people in Malaysia. The poor performance of teams could be mediating among the nature of the SQ and failure of detection and prevention of strategies. Bouwmans et al. (2019) examined the practices of teams and the performance of teams that contribute to processing of information and commitments. SQ nature should be analyzed from a rational preference for the SQ, as when the existing nature of affairs is equitably superior to the accessible opportunity. When imperfect information and lack of team performance are a powerful problem among the teams, controlling drugs in society could lead to the FDPS. Hsieh and Lin (2020) analyzed the team performance impacts that form an impact on the nature of the SQ and detection and prevention strategies. A large body of proof, however, shows that SQ nature, again and again, affects human decisions in Malaysia. SQ nature can also be described as psychological apathy, which assigns to a lack of interference of teams in the current state of affairs. Rau et al. (2018) discussed the crime prevention strategies with the relevance of drugs that are vulnerable to the neighborhoods of different countries. SQ prejudice has been attributed to a combination of loss of dissatisfaction and trust effects, two ideas relevant to the subject of strategies. The potential losses of changing from the SQ nature more heavily than the potential gains could help the governments in the prevention of drugs in the society of Malaysia. However, the SQ nature is managed even in the absence of gain/loss framing. Eaton and Mendonça (2019) enumerated the adaptation of process toward the poor or absolute team performance and its role toward the SQ nature and prevention and detection strategies. Loss aversion also causes more regret for action than inaction, and more regret is felt when a decision alters the SQ rather than preserving it. People are driven to do nothing or to keep current and past decisions as a result of various influences working together to benefit the SQ.

**H3:** PTP significantly and positively mediates the relationship between SQ nature and failure of detection and prevention of strategies.

Every leader who wishes to take prominence in the respective context needs to challenge the nature of resistance toward innovation (Chien et al., 2021b). It is clear that the system and management want the leaders and employees of Malaysia to protest against the people who are creating resistance toward the innovation. Guchait et al. (2020) narrated the impacts of error management of controls due to the team performance that mediates between strategies and innovation. Most of the leaders in the public get agitated due to PTP about the concept of change administration and renewal in search of the next big stuff. They appreciate reasoning about the boundless prospects of controlling drugs. Dakka (2020) examined the relationship between the diversity of resistance, innovation, and competition that impacts the strategies for the detection and prevention of drugs. Many of their team workers in turn are confident that their leaders will change their mentality from simply handling the rise and maintaining the nature of detection and prevention strategies. Timbang et al. (2019) established the opportunities that are important for the detection and prevention of drugs prominent in creating disease. The organization does not enable change and the leaders’ excitement fades very quickly when faced with the strategies for the detection and prevention of drugs in Malaysia. This is exactly how the system and its leaders get stuck in the resistance natures and we need them to be unstuck. Kindarto et al. (2020) assessed the role of government and leadership styles toward the team performance that asserts a critical role over the competence of strategies and innovation. Most governments and administrations are too afraid to do the elimination of resistance toward innovation. PTP inserts its mediating role among the resistance to innovation and strategies toward the detection and prevention of drugs. The mediating impact of PTP is clear in the strategies that are required to be established for the prevention and detection of drugs.

**H4:** PTP significantly and positively mediates the relationship between RTIN and FDPS.

### Study Gaps

In addition, this study addresses that some gaps do exist in the literature, namely, (1) being one of the important and sensitive topics, such as drug controlling, although studied but still not reached its peak, (2) Hasan et al. (2019) worked on the policy reforms of the drug regulate practices in Asian economies, whereas this study works on drug control prevention strategies with mediation effect in Malaysian pharmaceutical industry, (3) Lim and Morris (2020) worked on the illicit drug along with the trade, whereas this study tests the drugs strategies associated with SQ nature, RTIN, and PTP in Malaysian drug industry, (4) Suárez and Clua-García (2021) worked on the drug usage policies along with human rights, whereas this study works on drugs but from detection and prevention point of view along with the addition of mediation effect, i.e., PTP Malaysia, (5) the model is not tested before in Malaysia, hence this study checks the model in Malaysia perspective with new dataset, (6) Silooy and Wenda (2021) worked on the efforts to overcome the drugs in Malaysia, whereas this study works on drug detection and prevention strategies along with SQ nature, RTIN, and PTP in Malaysian pharmaceutical industry.

## Methodology

The research investigates the impact of the SQ and RTIN of drug control committee on the FDPS and also analyzes the mediating role of PTP among the SQ and RTIN of drug control committee and FDPS in Malaysia. This study has employed the primary data collection ways such as questionnaires to gather the data from selected respondents. This study has taken SQ with six items from the study by Engelke et al. (2019) and RTIN with five items taken from the study by Mani and Chouk (2018) as the predictive variable. In addition, this article has also taken the PTP as the mediating variable, with five items taken from the study. Finally, this research has used the FDPS as the dependent variable that has four items taken from the study by Wang et al. (2019).

These surveys were sent to the respondents using mail and personal visits. The members of the drug control committees in Malaysia are the respondents. The respondents were selected using simple random sampling. Thus, the researchers have sent around 630 surveys to the respondents, but only 357 were returned and used for analysis after a few weeks. These surveys represent about a 56.67% rate of response. Moreover, the researchers also applied the SPSS-AMOS to check the association among variables and testing of hypotheses. This tool is considered the best tool for primary data analysis. In addition, it also operates perfectly when the researchers adopt large datasets or complex modes. The model of the study is given in Figure 2.

**FIGURE 2:** Theoretical model.

## Research Findings

The research investigates the impact of the SQ and resistance to the innovative nature of the drug control committee on the FDPS and also analyzes the mediating role of PTP among the SQ and resistance to the innovative nature of the drug control committee and the FDPS in Malaysia. This study has employed the average variance extracted (AVE) to check the convergent validity. The statistics exposed that the AVE values are larger than 0.50 and exposed valid convergent validity. In addition, this article has also employed composite reliability (CR) to check the reliability, and the statistics exposed that the values of CR are larger than 0.70 and exposed significant reliability. The results also exposed that the factor loadings are more than 0.40, which is the indication of valid content validity. Table 1 shows the above mentioned figures.

**TABLE 1:** Convergent validity.

Constructs	Items	Loadings	CR	AVE
*Status quo*	SQ6	0.624	0.889	0.584
	SQ5	0.643		
	SQ4	0.604		
	SQ3	0.619		
	SQ2	0.981		
	SQ1	0.995		
Resistance to innovation nature	RTIN5	0.645	0.843	0.527
	RTIN4	0.527		
	RTIN3	0.639		
	RTIN2	0.860		
	RTIN1	0.892		
Poor team performance	PTP5	0.807	0.945	0.775
	PTP4	0.923		
	PTP3	0.975		
	PTP2	0.815		
	PTP1	0.870		
Failure of detection and prevention strategies	FDPS4	0.923	0.783	0.513
	FDPS3	0.946		
	FDPS2	0.405		
	FDPS1	0.380		

This study has employed the Fornell Larcker to check the discriminant validity and the statistics exposed that the first value in the column is higher than the other values that exposed a stronger association with the variable itself than other and exposed valid discriminant validity. Table 2 shows the above mentioned figures.

**TABLE 2:** Discriminant validity.

	FDPS	SQ	RTIN	PTP
FDPS	0.716			
SQ	0.531	0.764		
RTIN	0.615	0.435	0.726	
PTP	0.385	0.468	0.504	0.880

The results of the direct path revealed that the SQ and RTIN of the drug control committee have a positive association with the FDPS in Malaysia and accept H1 and H2. Table 3 shows the above mentioned Figure 3.

**TABLE 3:** Direct path.

Relationships			Beta	S.E.	C.R.	*P*
Poor team performance	←	*Status quo*	0.409	0.054	7.597	***
Poor team performance	←	Resistance to innovation nature	0.283	0.05	5.626	***
Failure of detection and prevention strategies	←	*Status quo*	0.362	0.047	7.629	***
Failure of detection and prevention strategies	←	Resistance to innovation nature	0.461	0.043	10.744	***
Failure of detection and prevention strategies	←	Poor team performance	0.086	0.043	1.987	0.047

***Show significant at 1%.

**FIGURE 3:** Measurement model assessment.

The findings of mediation analysis also exposed that PTP significantly mediates between SQ and RTIN of drug control committee and FDPS in Malaysia and accept H3 and H4. Table 4 shows the above mentioned Figure 4.

**TABLE 4:** Mediation analysis.

	SQ		RTIN	
		
	Beta	*P*-Values	Beta	*P*-Values
Total effects	0.453	0.000	0.254	0.000
Direct effects	0.292	0.023	0.282	0.000
Indirect effects	0.325	0.003	0.022	0.013

**FIGURE 4:** Structural model assessment.

## Discussion

The results indicated that the SQ nature of the drug control committee member has a positive impact on the FDPS of the committee related to the drug control in the society. This outcome indicated that the SQ members in the committee are not active to adopt new changes and are also not involved in the motivation process of drug-addicted individuals, which is the reason for the failure of their detection and prevention strategies to control the drug addiction people in the society. This outcome is similar to the study by Atkinson (2011) which also indicated that the SQ nature of the drug control committee member has a positive impact on the failure of their detection and prevention strategies. In addition, this result is also in line with the study by McCloskey et al. (2014) which also investigated that the SQ nature of the drug control committee member has a positive impact on the failure of their detection and prevention strategies. Because the SQ members are not active in the motivation process of drug-addicted individuals, that is the reason for the failure of their detection and prevention strategies to control the drug-addicted people. This finding is also the same as the findings of Barocas et al. (2022) which also examined that the members who are SQ in nature are not active in their operations and are considered very lazy in adopting and implementing new strategies, which is the reason of the failure of their detection and prevention strategies to control the drug-addicted people. The article results related to the SQ nature of the committee have a positive impact on the failure of drug control committee strategies, and this result is matched with the study by Del Pozo and Beletsky (2020) which also exposed that if the nature of the committee was SQ, then it leads toward the failure of drug control committee strategies in the country.

The findings also exposed that the RTIN in the member of the drug control committee also has a positive impact on the failure of their detection and prevention strategies to control the drug-addicted people. Thus, this output revealed that if the members of the drug control committee are not willing to adopt the innovation to control the drug-addicted people, then they fail to implement the detection and prevention strategies to control the drug-addicted people. This outcome is similar to the study by Dheda et al. (2017) which also investigated that the RTIN in the member of the drug control committee also has a positive impact on the failure of their detection and prevention strategies to control the drug-addicted people. Moreover, this result is also the same as the study by Robert (2011) which also revealed that the RTIN of drug control committee members has a positive impact on the failure of their detection and prevention strategies. Because the drug control committee members are unwilling to adopt the innovation to control the drug-addicted people, they fail to implement the detection and prevention strategies to control the drug-addicted people. This outcome is also in line with the study by Gandhi et al. (2010), which also exposed in the study that the RTIN among drug control committee members positively impacted the failure of their detection and prevention strategies to control the drug-addicted people. The research has examined that the RTIN of the committee has a positive impact on the failure of drug control committee strategies, and this result is in line with the study by Löscher et al. (2020) which also revealed that if the committee has RTIN, then it leads toward the failure of drug control committee strategies to control the drug-addicted individuals.

The results also indicated that the PTP significantly and positively mediates the association of the SQ nature of the drug control committee member and the FDPS of the committee related to the drug control in the society. This outcome exposed that if the drug control committee member has an SQ nature, they are not willing to adopt changes and produce PTP that leads to the FDPS of the committee related to the drug control. This outcome is similar to the study by Li and Shui (2015) which also investigated that the SQ nature of the employees leads them to PTP effect of the FDPS of the committee related to the drug control. In addition, this result is also in line with the study by Schaltegger and Csutora (2012) which indicated that PTP is the outcome of the SQ nature of the drug control committee member that leads to the FDPS of the committee.

The findings also indicated that the PTP significantly and positively mediates the association of RTIN of the drug control committee members and the FDPS of the committee related to the drug control in the society. This output revealed that if the members of the committee are not willing to adopt the innovation in the processes, then they fail to improve the performance of the team, also have an adverse effect, and also fail in the implementation of detection and prevention strategies of the committee to control the drug addiction people. This outcome is matched with the study by Hartono and Kusumawardhani (2019) which also investigated that the PTP is the outcome of the RTIN of the drug control committee members that leads to the FDPS of the committee to control the drug addiction people. In addition, this result is also in line with the study by Oreg (2018) which also examined that if the committee member is not willing to adopt the innovation, then they fail to improve the team performance and also have an adverse effect and fail in the implementation of detection and prevention strategies to control the drug addiction people. The research has also examined that the RTIN leads toward PTP and also moves toward the failure of drug control committee strategies, and this result is similar to the study by Liu et al. (2019) which also revealed that if the committee has RTIN, then it leads toward PTP and also moves toward the failure of drug control committee strategies.

### Theoretical Contributions

This article has some theoretical contributions and also has some practical implications. This study contributes to the literature on the SQ nature and FDPS of drug control committees. In addition, this research has also contributed to the existing literature on resistance to innovation and FDPS of drug control committees. Moreover, this study has significantly contributed to the existing literature by providing the literature on mediating role of PTP among the association of SQ nature and FDPS and resistance to innovation and FDPS. The investigation of mediating role of PTP is one of the first attempts.

### Practical Implications

In addition, this study provides help to the new researchers who want to examine this area in the future. This study guides policymakers in developing policies that eliminate the SQ nature and motivate the committee to adopt innovation that enhances team performance and success of detection and prevention strategies in Malaysia. This study also guides the policy implementation authorities that they should focus on the members of the committee regarding their nature and way of dealing with drug-addicted people. Finally, this article guides the drugs control institutions that they must check the nature of their drug control committee that significantly affected their strategies to control the drug-addicted people in the country.

### Limitations and Future Directions

This article has some limitations that would be the directions for the upcoming literature. This study has taken only two predictors, such as SQ nature and RTIN, to predict the FDPS of the drug control committee and ignore other factors. This article suggested that future articles should add more factors to predict the drug control committee’s FDPS. In addition, this article has taken the PTP as a mediating variable and ignored the moderating variable in the study and suggested that future studies focus on moderating variables in the context. Moreover, this article has examined the drug control committees of Malaysia and ignored the other countries and recommended that upcoming studies should add more countries to expand the scope of the study. Finally, this article has used the SPSS-AMOS and also recommended that future studies should also use the smart-PLS for the analysis purpose.

## Data Availability Statement

The original contributions presented in this study are included in the article/supplementary material, further inquiries can be directed to the corresponding author.

## Author Contributions

The author confirms being the sole contributor of this work and has approved it for publication.

## Conflict of Interest

The author declares that the research was conducted in the absence of any commercial or financial relationships that could be construed as a potential conflict of interest.

## Publisher’s Note

All claims expressed in this article are solely those of the authors and do not necessarily represent those of their affiliated organizations, or those of the publisher, the editors and the reviewers. Any product that may be evaluated in this article, or claim that may be made by its manufacturer, is not guaranteed or endorsed by the publisher.
